This article has been retracted.

# Loureirin A Exerts Antikeloid Activity by Antagonizing the TGF-*β*1/Smad Signalling Pathway

**DOI:** 10.1155/2022/8661288

**Published:** 2022-07-15

**Authors:** Hui Ma, Xingwu Duan, Runtian Zhang, Hang Li, Yang Guo, Ye Tian, Min Huang, Guangshan Chen, Zi Wang, Lingling Li

**Affiliations:** ^1^Department of Dermatology, Beijing Hospital of Traditional Chinese Medicine, Capital Medical University, 23 Back Street, Art Museum, Dongcheng District, Beijing 100010, China; ^2^Department of Dermatology, Dongzhimen Hospital, Beijing University of Chinese Medicine, No. 5 Shipping Warehouse, Dongcheng District, Beijing 100700, China; ^3^Department of Dermatology, Peking University First Hospital, No. 8 Xishiku Street, Xicheng District, Beijing 100034, China

## Abstract

It has been recently shown that loureirin A (LA), a major active component of resina draconis, might be effective in the prevention and treatment of liver fibrosis. We examined whether LA could inhibit the formation of keloids. To investigate the pharmacological effects of loureirin A on keloid formation and the underlying mechanisms. CellTiter-Blue viability assays were used to examine the proliferation of keloid fibroblasts (KFs) that were treated with LA. Fibroblast migration was evaluated using a cell migration assay. Immunofluorescence staining was used to measure the expression of *α*-SMA in KFs. RT-qPCR was used to evaluate the mRNA expression of Col-I, Col-III, *α*-SMA, Bax, and Caspase-3, while Western blotting was used to evaluate the protein expression of Col-I, Col-III, *α*-SMA, Bax, Caspase-3, p-Smad2, and p-Smad3. LA inhibited the proliferation of KFs and suppressed the migration and TGF-*β*1-induced myofibroblast differentiation of KFs. In addition, LA downregulated the mRNA and protein levels of Col-I, Col-III, and *α*-SMA while promoting the mRNA and protein levels of Bax and Caspase-3. Moreover, LA downregulated the protein levels of p-Smad2 and p-Smad3 in cultured TGF-*β*1-treated KFs ex vivo. These results show that LA has an antikeloid effect on KFs by suppressing the TGF-*β*1/Smad signalling pathway. Our findings suggest that LA may be a potential candidate drug for the prevention and treatment of keloids.

## 1. Introduction

Keloids are benign dermal fibroproliferative growths that are unique to humans [1]. Keloid tissue is characterized by an overabundant accumulation of extracellular matrix (ECM), which consists of collagen I (Col-I) and collagen III (Col-III), in the dermis and subcutaneous tissue that extends beyond the confines of the original wound site [2, 3]. Keloids represent a form of abnormal wound healing in genetically susceptible individuals and are common in dark-pigmented ethnicities with up to 15% of that population at risk [4]. Clinically, keloids not only affect skin appearance but also affect the physical and psychological health of patients. Currently, there are multiple treatment modalities, such as intralesional steroid injection, surgery, radiation, and laser therapy, as well as combination therapy consisting of several methods mentioned above [3]. However, the optimal option has not been established and further research is needed.

Genetically, several lines of evidence suggest that multiple genetic loci are involved in susceptibility to keloids [5, 6]. Pathologically, it is widely believed that fibroblasts and myofibroblasts are the key cells related to keloid formation through the production of ECM [7]. Moreover, melanocytes and keratinocytes both play important roles; melanocytes contact or interact with fibroblasts after basal membrane injury to promote the proliferation of fibroblasts and the deposition of collagen [8], while keratinocytes can secrete transforming growth factor-beta (TGF-*β*). Keratinocyte-fibroblast interactions also regulate myofibroblast transformation [9]. Keloid formation is also the result of excessive expression of growth factors and cytokines, such as TGF-*β*, platelet-derived growth factor subunit B (PDGF-B), vascular endothelial growth factor (VEGF), and tumour necrosis factor-*α* (TNF-*α*) [10, 11]. Related studies on cytokines have shown that the overexpression of TGF-*β*1 or TGF-*β*2 and decreased expression of TGF-*β*3 exert a prominent driving force on the formation of keloidal scars and create an environment that activates fibroblasts [12]. In terms of fibrotic signalling pathways, several pathways are involved in keloid formation, including the mitogen-activated protein kinase (MAPK), insulin-like growth factor-I (IGF-I), integrin, and TGF-*β*1/Smad pathways, of which the TGF-*β*1/Smad pathway is thought to be the most critical [13]. Although many studies on keloids have been performed, the accurate pathophysiological mechanism of keloid formation is still unclear. Keloid formation is a complex process and involves a network of cells, cytokines, molecules, and signalling pathways [12].

The ethnomedicine Resina Draconis (RDEE) is a kind of resinous medicine extracted from the tree stem of *Dracaena cochinchinensis* and is commonly prescribed to invigorate blood circulation to treat traumatic injuries, blood stasis, and pain [14]. Modern pharmacological studies have shown that this resinous medicine has anticoagulation, anti-inflammatory, and antitumor effects and can promote skin repair activities. Various compounds have been isolated from the plant, including loureirin A, loureirin B, loureirin C, cochinchinenin, socotrin-4′-ol, 4′,7-dihydroxyflavan, 4-methylcholest-7-ene-3-ol, ethylparaben, resveratrol, and hydroxyphenol [15]. Loureirin A (LA) is a known major active component of the ethanolic extract of RDEE. A recent study showed that LA could inhibit the proliferation of hepatic stellate cells and inhibit the secretion of alpha-smooth muscle actin (*α*-SMA) and TGF-*β*1, which suggests that LA might have potential antifibrosis efficacy [16]. However, whether LA could also treat keloids has not been determined. In this study, we clarified the pharmacological effects of LA on keloid formation and the underlying mechanisms to provide a novel treatment strategy for keloids.

## 2. Materials and Methods

### 2.1. Tissue Samples and Chemical Reagents

Keloid scar specimens were surgically obtained from the breasts of four Chinese patients (male, 25 years old; male, 28 years old; female, 3 years old; female, 35 years old) with an average age of 30 years. The patients received no treatment before the surgical excision, which was performed in the Department of Dermatology at Peking University First Hospital, Beijing, China. All experiments were approved by the Ethics Committee of Dongzhimen Hospital, Beijing University of Chinese Medicine (protocol no: DZMEC-KY-2019-174). Written informed consent was provided by each patient.

LA (Bioruler, US) was dissolved in 100% dimethyl sulfoxide (DMSO, Sigma, US) to a stock concentration of 100 mg/ml and stored under light-protected conditions at −20°C. Animal-free recombinant human TGF-*β*1 (Proteintech, US) was dissolved in sterile 4 mM HCl with 0.1% bovine serum albumin (BSA, Invitrogen, US) and yielded a final stock concentration of 10 *μ*g/ml. On the day of use, the stock solutions were directly diluted to the desired concentration with 10% foetal bovine serum (FBS, Gibco, US) prepared with Dulbecco's modified Eagle's medium (DMEM, Gibco, US). The final concentration of DMSO did not exceed 0.1% (v/v) in all experiments.

### 2.2. Cell Culture

Keloid tissues were excised under local anaesthesia and collected in a 50 ml centrifuge tube; the tissues were washed three times in phosphate buffer solution (PBS, Gibco, US) containing 1% penicillin and 1% streptomycin for 5 min each time. Afterward, the samples were trimmed with a scalpel to remove the *epidermis* and excessive adipose tissues, and the remaining dermis was minced into small pieces approximately 1 mm^3^ in size. Then, the small pieces were uniformly incubated in 20% FBS in a vertical 25 ml culture bottle for 4 h at 37°C in a humidified atmosphere of 5% CO_2_, after which the bottle was gently laid flat. Next, 2 ml of nutrient medium was added the following day, and the medium was changed every four days. The fibroblasts grew out of the tissues after 3–5 days of culturing. Primary KFb cells were collected and maintained at 37°C in a humidified atmosphere of 5% CO_2_, and subcultured using PBS/0.05% trypsin-ethylenediaminetetraacetic acid (EDTA, Gibco, US) when the cells reached 80–90% confluence. The fibroblasts used in all experiments were from the 3^rd^ to 5^th^ passages.

### 2.3. CellTiter-Blue Viability Assay

Human primary keloid fibroblasts (KFs) were seeded in 96-well plates at 1000 cells per well in 100 *μ*l of medium and incubated overnight at 37°C in a humidified atmosphere of 5% CO_2_. Afterward, the cells were treated with LA (50, 30, and 10 *μ*g/ml), TGF-*β*1 (40, 20, and 10 ng/ml), or 10% FBS (control) and then analysed with CellTiter-Blue reagent (Promega, US) at 24, 48, and 72 h. Briefly, at each time point, 20 *μ*l of sterile CellTiter-Blue reagent was added to each well and incubated for 4 h at 37°C, and then the medium was harvested to measure the fluorescent signal at 560 Ex/590 Em using a microplate reader (Thermo Scientific, US). All assays were performed in triplicate and repeated using four independent cell samples (*n* = 4, 12 samples). The percentage of the cell inhibition/proliferation rate was calculated with the following formulas: cell inhibition rate = 1-experimental well/control well × 100%; cell proliferation rate = (experimental well/control well-1) × 100% [4].

### 2.4. Cell Migration Assay

An in vitro scratch wound assay was used to evaluate cell migration [17]. KFs were seeded in 6-well plates at a density of 2 × 10^5^ cells per well and incubated overnight (37°C, 5% CO_2_). When the cells reached 90% confluence, the cell monolayer was scratched with a sterile 5 ml pipette tip and incubated in culture medium containing TGF-*β*1 (40 ng/ml), LA (50 *μ*g/ml) + TGF-*β*1 (40 ng/ml) or 10% FBS (control) for 48 h. Photographs were taken at 0 and 48 h after scratching. The photographed area was quantified with Image-Pro Plus 6.0 software (IPP 6.0). The results are presented as the percentage of the scratched area filled by keloid cells within 48 h. The data were acquired from five randomly selected high-power fields.

### 2.5. Immunofluorescence Staining

KFs were seeded into 15 mm glass bottom cell culture dishes at a density of 4.0 × 10^4^ cells per well with different drug treatments for 48 h. After being washed with PBS, the cells were fixed with 4% paraformaldehyde for 15 min, permeabilized with 0.1% Triton X-100 (Solarbio, China) for 15 min, blocked with 5% BSA at room temperature for 1 h, and incubated with anti-*α*-SMA antibody (Proteintech, US) overnight at 4°C. On the next day, the cells were incubated with CoraLite594-conjugated goat anti-rabbit IgG (*H* + *L*) secondary antibodies (Proteintech, US) for 1 h at room temperature in the dark. DAPI (Sigma-Aldrich, US) was used for nuclear staining. Images were obtained using a TCS SPE confocal microscope (Leica, GER). Images were analysed by IPP 6.0 [18].

### 2.6. Reverse Transcription Quantitative Real-Time Polymerase Chain Reaction (RT-qPCR)

Total RNA was extracted from human keloid-derived fibroblasts using a RNeasy mini kit (Qiagen, GRE). The purity of the obtained RNA was determined by the A_260_/A_280_ ratio. RNA samples (1.0 *μ*g) were reverse transcribed with the PrimeScriptRT reagent kit (Takara, Japan). The resulting cDNA was then amplified by using the SYBR Premix Ex Taq kit (Takara, Japan) with primer pairs that were specific to the target genes. The sequences for primers are as follows: Col-I, 5′-CAGCAGATCGAGAACA.

TCC-3′ (forward) and 5′-TCCAGTACTCCCACTCTTC-3′ (reverse); Col-III, 5′-GGAGCTGGCTACTTCTCGC-3′ (forward) and 5′-GGGAACATCCTCCTTCAAC.

AG-3′ (reverse); *α*-SMA, 5′-CATCATGCGTCTGGATCTG-3' (forward) and 5′-TCACGCTCAGCAGTAGTA-3′ (reverse); Bax, 5′-CCCGAGAGGTCTTTTTCCGA.

G-3′ (forward) and 5′-CCAGCCCATGATGGTTCTGAT-3′ (reverse); Caspase-3, 5′-AGAGGGGATCGTTGTAGAAGTC-3′ (forward) and 5′-ACAGTCCAGTTCT.

GTACCACG-3′ (reverse); and GAPDH: 5′-CAGGAGGCATTGCTGATGAT-3′ (forward) and 5′-GAAGGCTGGGGCTCATTT-3′ (reverse). The mRNA expression was normalized to that of GAPDH. Fold changes in mRNA were analysed using the 2^−ΔΔCt^ method [19].

### 2.7. Western Blotting

KFs were treated as previously described, and total proteins were extracted using RIPA lysis buffer and quantified with a bicinchoninic acid assay kit (Sigma-Aldrich, US). Equal amounts of protein were separated by SDS-PAGE and then transferred onto PVDF membranes (Millipore, MA). After blocking with 5% nonfat milk, the membranes were incubated with the appropriate primary antibodies overnight at 4°C. On the following day, the membranes were washed three times with TBST (Solarbio, US) and then incubated with species-matched secondary antibodies. The membrane-bound proteins were detected using an enhanced chemiluminescence detection kit (Pierce, US) and quantified using ImageJ software. The primary antibodies used were as follows: (i) p-Smad2 (SAB4301424) and p-Smad3 (SAB4301416) (all from Sigma-Aldrich, US); (ii) Smad2 (12570-1-AP), Smad3 (66516-1-Ig), Col-I (14695-1-AP), Col-III (22734-1-AP), *α*-SMA (55135-1-AP), Bcl-2 (12789-1-AP), Bax (50599-2-Ig), caspase-3 (19677-1-AP) and *β*-actin (20536-1-AP) (all from Proteintech, US). *β*-Actin served as an internal control [20].

### 2.8. Statistical Analysis

All data are presented as the mean ± SD. Statistical significance was determined by one-way analysis of variance (ANOVA) for differences among multiple comparisons (>2 groups) using SPSS 20.0 software (Chicago, US). *P* values < 0.05 were considered statistically significant.

## 3. Results

### 3.1. Loureirin A Inhibits and TGF-*β*1 Promotes KF Proliferation

We first selected the optimal treatment time for LA (chemical structure is shown in Figure 1(a)) and TGF-*β*1 by CellTiter-Blue cell viability assays. The results showed that LA inhibited cell proliferation while TGF-*β*1 promoted cell proliferation, and the optimal stimulation time was 48 h (Figures 1(b) and 1(c)). Then, at 48 h, the optimal concentrations of LA and TGF-*β*1 to stimulate the mRNA expression of Col-I, Col-III, and *α*-SMA were determined by RT-qPCR. LA downregulated and TGF-*β*1 upregulated the mRNA expression of Col-I, Col-III, and *α*-SMA in a dose-dependent manner (Figures 1(d) and 1(e)). Moreover, the optimal concentrations of LA and TGF-*β*1 were 50 *μ*g/ml and 40 ng/ml, respectively. Therefore, these conditions were used in subsequent experiments.

### 3.2. Loureirin A Suppresses the Migration of TGF-*β*1-Induced KFs

As scar formation is often accompanied by enhanced migration of dermal fibroblasts [21], we wondered whether LA could inhibit the migration of KFs in vitro. As shown in Figures 2(a) and 2(b), the migration of KFs in the TGF-*β*1 (40 ng/ml) group was enhanced compared with that in the control group. After 48 h of culture, 41.2 ± 1.5% of the scratched area was filled after TGF-*β*1 treatment. In contrast, the enhanced migration of KFs by TGF-*β*1 was evidently abrogated by LA (50 *μ*g/ml), and only 30.7 ± 2.5% of the scratched area was filled (*F* = 31.35, LA + TGF-*β*1 vs. TGF-*β*1, *P* < 0.01). Thus, LA could suppress the migration of TGF-*β*1-induced KFs.

### 3.3. Loureirin A Inhibits TGF-*β*1-Induced Differentiation of KFs into Myofibroblasts

Myofibroblasts are the main cells responsible for scar contraction through the expression of *α*-SMA. Fibroblasts can be transformed into myofibroblasts after injury and play a crucial role in the formation of keloids [22–24]. The expression of *α*-SMA, a marker of myofibroblasts, in KFs exposed to control (10% FBS), TGF-*β*1 (40 ng/ml) or LA (50 *μ*g/ml) + TGF-*β*1 (40 ng/ml) for 48 h was measured by immunofluorescence staining. As shown in Figures 3(a) and 3(b), the expression of *α*-SMA (red) following treatment with TGF-*β*1 was apparently enhanced compared with that in the control group; however, this effect was markedly attenuated by LA (*F* = 221.90, TGF-*β*1 vs. control, *P* < 0.01; LA + TGF-*β*1 vs TGF-*β*1, *P* < 0.01). These results demonstrated that LA could inhibit TGF-*β*1-induced myofibroblast differentiation of KFs in vitro.

### 3.4. Loureirin A Downregulates the Expression of Col-I, Col-III, and *α*-SMA in TGF-*β*1-Induced KFs

Keloid tissue is mostly characterized by an overabundant accumulation of ECM, which is composed of disorganized Col-I and Col-III and excess myofibroblasts [25]. Surprisingly, in keloids, collagen synthesis was approximately 20 times higher than that in normal, unscarred skin [26]. To investigate the effect of LA on the expression of ECM, we measured the mRNA and protein levels of Col-I, Col-III, and *α*-SMA in KFs by RT-qPCR and Western blotting, respectively. KFs were divided into three groups: control (10% FBS), TGF-*β*1 (40 ng/ml) and LA (50 *μ*g/ml) + TGF-*β*1 (40 ng/ml). The results (Figures 4(a) and 4(b)) showed that TGF-*β*1 treatment notably increased the mRNA and protein levels of Col-I, Col-III, and *α*-SMA, which were dramatically inhibited by LA (Col-I: *F* = 370.35, LA + TGF-*β*1 vs TGF-*β*1, *P* < 0.01; Col-III: *F* = 133.27, LA + TGF-*β*1 vs TGF-*β*1, *P* < 0.05; *α*-SMA: *F* = 413.68, LA + TGF-*β*1 vs TGF-*β*1, *P* < 0.01). These data suggested that LA might exert an antikeloid effect by reducing the synthesis of ECM.

### 3.5. Loureirin A Promotes Apoptosis in TGF-*β*1-Induced KFs

It is believed that the proliferation and apoptosis of KFs should be balanced; otherwise, ECM deposition may be delayed or result in excessive scarring. Researchers have demonstrated a significantly lower rate of apoptosis in keloidal fibroblasts than in normal skin fibroblasts [27]. To further investigate the effect of LA on KF apoptosis, we next measured the mRNA and protein expression of Bax and Caspase-3 in KFs. KFs were divided into three groups: control, LA (50 *μ*g/ml) + TGF-*β*1 (40 ng/ml), and TGF-*β*1 (40 ng/ml). As shown in Figures 5(a) and 5(b), TGF-*β*1 had no obvious effect on the mRNA and protein expression levels of these genes, whereas the mRNA and protein expression levels of Bax and Caspase-3 were dramatically increased when cells were treated with LA + TGF-*β*1 (Bax: *F* = 82.34, LA + TGF-*β*1 vs TGF-*β*1, *P* < 0.01; Caspase-3: *F* = 124.75, LA + TGF-*β*1 vs TGF-*β*1, *P* < 0.01). Taken together, these results indicated that LA could promote apoptosis in TGF-*β*1-induced KFs.

### 3.6. Loureirin A Suppresses the TGF-*β*1/Smad Signalling Pathway in TGF-*β*1-Induced KFs

To elucidate the underlying molecular mechanism of LA-mediated proliferation, apoptosis, and ECM synthesis in KFs, the protein expression ratios of p-Smad2/Smad2 and p-Smad3/Smad3 were examined. KFs were divided into three groups: control, LA (50 *μ*g/ml) + TGF-*β*1 (40 ng/ml), and TGF-*β*1 (40 ng/ml). As shown in Figure 6, TGF-*β*1 treatment notably increased the expression of these proteins in KFs, which was dramatically inhibited by LA (p-Smad2/Smad2: *F* = 7.03, LA + TGF-*β*1 vs TGF-*β*1, *P* < 0.05; p-Smad3/Smad3: *F* = 26.40, LA + TGF-*β*1 vs TGF-*β*1, *P* < 0.05). These results showed that LA suppressed the TGF-*β*1/Smad signalling pathway in TGF-*β*1-induced KFs.

## 4. Discussion

In the present study, the pharmacological effects of LA on keloid-derived fibroblasts were first investigated, and the potential underlying mechanism was clarified. Keloids are known to contain a large number of highly proliferative fibroblasts, which synthesize elevated levels of ECM that consists of Col-I and Col-III [3]. Although many cytokines are involved in the formation of keloids, TGF-*β*1 is considered one of the most potent stimulators that can induce fibroblast chemotaxis and proliferation, promote the trans-differentiation of fibroblasts into myofibroblasts, and induce ECM synthesis [28, 29]. Therefore, we further examined the effects of LA on TGF-*β*1-stimulated KFs. CellTiter-Blue cell viability assays showed that LA could inhibit the proliferation of KFs, and the optimal concentration of LA was 50 *μ*g/ml. Cell migration assays showed that LA restrained the migration of TGF-*β*1-induced KFs. Immunofluorescence staining showed that LA inhibited TGF-*β*1-induced myofibroblast differentiation of KFs in vitro. Moreover, our results demonstrated that LA prominently downregulated the TGF-*β*1-induced mRNA and protein levels of Col-I, Col-III, and *α*-SMA.

Furthermore, aberrant cell apoptosis is crucial in the formation of keloids. The dysregulation of apoptosis and the proliferation of fibroblasts in keloids results in massive secretion of collagen and ECM [30, 31]. Therefore, the expression of the proapoptotic molecules Bax and Caspase-3 was measured to evaluate the effect of LA on the apoptosis of TGF-*β*1-stimulated KFs [32, 33]. Our results showed that LA dramatically increased the mRNA and protein expression levels of Bax and Caspase-3 compared with that of TGF-*β*1, which indicated that LA could promote apoptosis in TGF-*β*1-induced KFs.

Although the fundamental molecular mechanism of keloid formation remains unclear, the TGF-*β*1 pathway is strongly believed to be a major player in keloid pathogenesis [34]. TGF-*β*1 transmits its signals mainly via the Smad family. TGF-*β*1 binds with TGF-*β* receptor II and then activates TGF-*β* receptor I on the cell membrane. Activated TGF-*β* receptor I phosphorylate receptor-regulated Smads (Smad2 and Smad3), and then the engagement of phosphorylated Smad2/3 with Smad4 allows for translocation into the nucleus and regulation of target gene transcription [29, 35]. In this study, we examined the phosphorylation levels of Smad2 and Smad3 to explore the potential underlying mechanism. The results showed that the protein levels of p-Smad2 and p-Smad3 were apparently downregulated (Figure 6), indicating that the inhibitory effects of LA on TGF-*β*1-induced KFs might occur through the TGF-*β*1/Smad pathway. Indeed, in addition to this pathway, crosstalk among cellular signalling pathways underlying keloid pathogenesis has been widely studied. For example, sorafenib exerts antikeloid activity by antagonizing the TGF-*β*/Smad and MAPK/ERK signalling pathways, leading to new approaches for future therapeutic improvements [21]. Certainly, more detailed investigations will be performed to verify the potential application of LA in the future.

Similarly, it has been shown that loureirin B (LB), another major component of REDD, could suppress fibroblast proliferative activity and dose-dependently downregulate both the mRNA and protein levels of Col-I, Col-III, and *α*-SMA in HS fibroblasts; moreover, LB not only suppressed the activation of Smad2 and Smad3 but also downregulated p-ERK and p-JNK in TGF-*β*1-stimulated fibroblasts, suggesting that LB could inhibit scar formation via the TGF-*β*/Smad and ERK/JNK signalling pathways [14, 36]. Thus, as the main components of REDD, both LA and LB may be effective in the prevention of pathological scars in vitro. The limitation of this study is that the LB Group was not set up to evaluate the difference in the efficacy of LA and LB in inhibiting keloid. Therefore, which is more effective among LA and LB is a new issue worth further study.

In terms of clinical application, compared with local injection or combined with CO_2_ dot array laser therapy, the absorption rate of external coating alone is much lower. Therefore, it is hoped that the absorption of monomer can be gradually improved through follow-up studies to improve its clinical efficacy.

## 5. Conclusions

Taken together, these in vitro findings demonstrated that LA could regulate the balance between KF proliferation and apoptosis, inhibit cell migration, and suppress collagen synthesis through the TGF-*β*1/Smad signalling pathway in TGF-*β*1-induced KFs. Thus, the potential therapeutic value of LA for keloid treatment was revealed through preliminary, fundamental research. However, the precise underlying mechanism and clinical efficacy need further elucidation.

Thus, it is conceivable that modulating DKK3 expression may provide a new therapy for keloid treatment.

## Figures and Tables

**Figure 1:** Loureirin A inhibits and TGF-*β*1 promotes KF proliferation. (a) The chemical structure of LA. (b) KFs were divided into four groups treated with 50, 30, and 10 *μ*g/ml LA or 10% FBS as a control group for 24 h, 48 h, and 72 h. The CellTiter-Blue cell viability assay showed that LA inhibited cell proliferation. (c) KFs were divided into four groups and treated with 40, 20, 10 ng/ml TGF-*β*1 or 10% FBS as a blank control for 24 h, 48 h, and 72 h. The results showed that TGF-*β*1 promoted cell proliferation. (d, e) KFs were divided into four groups and treated with LA or TGF-*β*1 for 48 h. The RT-qPCR results showed the mRNA levels of Col-I, Col-III, and *α*-SMA. The data were normalized to the control and are presented as the mean ± SEM. ^*∗*^*P* < 0.05, ^*∗∗*^*P* < 0.01 compared with the control group. Each assay was performed in triplicate and repeated using four independent cell samples (*n* = 4, 12 samples).

**Figure 2:** Loureirin A suppresses the migration of TGF-*β*1-induced KFs. (a, b) KFs were seeded in 6-well plates and separated into three groups: control (10% FBS), TGF-*β*1 (40 ng/ml) and LA (50 *μ*g/ml) + TGF-*β*1 (40 ng/ml). The cell monolayer was scratched, and the filling of the scratched areas by migrated KFs was observed at 48 h postscratching and quantified using IPP software. The data are presented as the mean ± SEM. ^##^*P* < 0.01 compared with the control group. ^*∗∗*^*P* < 0.01 compared with the TGF-*β*1 group. Each assay was performed in triplicate and repeated using four independent cell samples (*n* = 4, 12 samples).

**Figure 3:** Immunofluorescence staining of *α*-SMA in TGF-*β*1-treated KFs. The expression of *α*-SMA (a) on the surface of the cell membrane. DAPI was used for nuclear counterstaining (b). The data are presented as the mean ± SEM. ^##^*P* < 0.01 compared with the control group, ^*∗∗*^*P* < 0.01 compared with the TGF-*β*1 group. Each assay was performed in triplicate and repeated using four independent cell samples (*n* = 4, 12 samples).

**Figure 4:** Loureirin A downregulates the expression of Col-I, Col-III, and *α*-SMA in TGF-*β*1-induced KFs. The mRNA and protein expression of Col-I, Col-III, and *α*-SMA were detected by RT-qPCR and Western blotting, respectively. (a) RT-qPCR and (b) Western blot results. The data are presented as the mean ± SEM. ^#^*P* < 0.05, ^##^*P* < 0.01 compared with the control group, ^*∗*^*P* < 0.05, ^*∗∗*^*P* < 0.01 compared with the TGF-*β*1 group. Each assay was performed in triplicate and repeated using four independent cell samples (*n* = 4, 12 samples).

**Figure 5:** Loureirin A promotes apoptosis in TGF-*β*1-induced KFs. The mRNA and protein expression of Bax and Caspase-3 were detected by RT-qPCR and Western blotting, respectively. (a) RT-qPCR and (b) Western blot results. The data are presented as the mean ± SEM. ^*∗∗*^*P* < 0.01 compared with the TGF-*β*1 group. Each assay was performed in triplicate and repeated using four independent cell samples (*n* = 4, 12 samples).

**Figure 6:** Loureirin A suppresses the TGF-*β*1/Smad signalling pathway in TGF-*β*1-induced KFs. The protein expression levels of p-Smad2 and p-Smad3 were detected by Western blotting. The data are presented as the mean ± SEM. ^*∗*^*P* < 0.05 compared with the TGF-*β*1 group. ^#^*P* < 0.05, ^##^*P* < 0.01 compared with the control group. Each assay was performed in triplicate and repeated using four independent cell samples (*n* = 4, 12 samples).

## Data Availability

The data used of this study are available from the corresponding author upon request.
